RETRACTED

# Diet and Lifestyle Impact on Rheumatoid Arthritis: A Comprehensive Review

**DOI:** 10.7759/cureus.48625

**Published:** 2023-11-10

**Authors:** Kartikey V Shekhar, Mrunmayee M Pathak, Gajanan Pisulkar

**Affiliations:** 1 Medical Education, Jawaharlal Nehru Medical College, Datta Meghe Institute of Higher Education and Research, Wardha, IND; 2 Orthopaedics, Jawaharlal Nehru Medical College, Datta Meghe Institute of Higher Education and Research, Wardha, IND

**Keywords:** synbiotics, essential fatty acids, foods, diets, rheumatoid arthritis

## Abstract

A systemic, inflammatory illness such as rheumatoid arthritis (RA) causes progressive cartilage and bone degradation in addition to joint involvement. Factors related to genetics and environment determine susceptibility to RA. In recent years, an increasing body of research has illuminated the pivotal role of diet and lifestyle in influencing the risk and progression of illnesses. Some nutrients, like polyunsaturated fatty acids, can combat inflammation. They also act as antioxidants, thus protecting against the onset of RA. Conversely, substances like salt and red meat have adverse effects, promoting the development and progression of RA through indirect mechanisms that impact gut microbiota and body composition. As we look ahead, potential supplementary therapies alongside the existing RA treatment regimen may manifest as specific dietary patterns and supplements. Promising candidates include the Mediterranean Diet (MD), vitamin D, and probiotics, which could potentially confer protective benefits. A poor level of education and low socioeconomic status, as well as smoking, an unhealthy diet, and obesity, have all been linked to an increased risk of RA in large epidemiological studies. Additionally, several lifestyle choices affect how well RA responds to antirheumatic medications. A worse treatment outcome is linked, among other things, to smoking, obesity, and insufficient physical activity. Therefore, RA sufferers must be urged to live a healthy lifestyle and eat well.

## Introduction and background

Rheumatoid arthritis (RA) is an inflammatory ailment known for its capacity to inflict significant damage upon synovial joints, often leading to profound disability and heightened mortality rates [1]. The etiology of RA is intricate, with genetic and environmental elements serving as critical determinants in its commencement and severity [1]. A well-established risk factor is a genetic predisposition supported by epidemiological data that illustrates an elevated vulnerability in individuals with a familial history of RA [2]. Gender and age also wield considerable influence, with women and middle-aged individuals being more frequently affected. Lifestyle choices, such as smoking, excessive consumption of red meat, lack of exercise, low intake of dietary fibers and essential fatty acids, consumption of alcohol, and gluten consumption, further augment the risk, while infectious agents like Epstein-Barr virus, retroviruses, and parvovirus B19 can potentially incite or exacerbate the condition [1,3]. Hormonal, dietary, socioeconomic, and ethnic aspects further contribute to the multifaceted nature of RA's pathogenesis. Importantly, many of these elements are interlinked, impacting the ailment's evolution and progression. Understanding the interplay between genetic and environmental factors is paramount in enhancing preventive measures, diagnosis, and management of RA [1].

RETRACTED

Among these factors, dietary choices and nutritional intake have been the subject of extensive research regarding their potential involvement in the onset and progression of autoimmune diseases [2]. Although some research has suggested that there may be a link between specific dietary patterns - especially when it comes to the amount of fruit, vegetables, and meat consumed and diseases like RA - the findings are still unclear. A growing amount of research has been conducted in recent years to examine the role nutrition and food may have in managing and preventing many illnesses, including RA [2,3]. When considering genetic and other lifestyle variables, the Mediterranean diet has a role in the reduced prevalence of RA in Southern Europe as opposed to Northern Europe and North America [4]. The main goals of this research are to investigate how nutrition and food affect the development of RA and to evaluate how nutritional choices can potentially influence the disease's activity [3,5].

## Review

Methodology

We performed a comprehensive search in the electronic databases PubMed, Medline, Embase, Google Scholar, and ResearchGate and an examination of the English-language literature. Inclusion criteria include peer-reviewed journals produced in English, articles published in the last 15 years, the full text of the publication; type of publication: review articles, systematic review, meta-analysis, or empirical studies published in peer-reviewed scientific journals; compliance with the combinations of keywords: synbiotics, essential fatty acids, human leukocyte antigen, elimination diet, rheumatoid arthritis. Exclusion criteria for the study encompass articles that don't provide the full text of the publication, are not in English, fall outside the specified publication types (review articles, systematic reviews, meta-analyses, or empirical studies in peer-reviewed scientific journals), involve malignancy or co-morbidities impacting the disease's presentation, present treatment protocols other than those under review. Key terms used for the search were "synbiotics"[all fields] or "essential fatty acids"[all fields] and "Human Leukocyte Antigen"[all fields] or "Elimination Diet"[Mesh terms] or "rheumatoid arthritis"[all fields]. The Preferred Reporting Items for Systematic Reviews and Meta-Analyses (PRISMA) method used in the research methodology are depicted in Figure 1.

RETRACTED

**Figure 1:** The selection process of articles used in this study. Preferred Reporting Items for Systematic Review and Meta-Analysis (PRISMA) flowchart for the keywords used in the literature review.

Years before the disease's clinical presentation, a multi-step process involving interactions between hereditary and environmental variables begins the pathogenesis of RA. The human leukocyte antigen (HLA) class II molecule is encoded on chromosome 6p21.3, the most important genetic risk locus linked to RA. A typical amino acid sequence known as the "shared epitope" (SE) is found at locations 70-74 in the third region of the DR-1 chain in several HLA-DRB1 alleles associated with seropositive RA [4]. In genetically susceptible people, environmental factors can compromise their endurance to autoantigen, such as citrullinated and carbamylated proteins. Long before any detectable symptoms appear, various environmental factors, including cigarette smoking, air pollution, exposure to dust, dietary habits, and susceptibility to infections, significantly contribute to developing autoantibodies and systemic autoimmune responses [5]. The pathophysiology of RA is supported by several important discoveries that point to the role of environmental, nutritional, reproductive, and lifestyle variables. For example, the fact that two-thirds of RA patients are female may indicate a potential function for female hormones. Furthermore, the incidence and age at the beginning of RA exhibit a discernible latitude gradient effect, and higher educational attainment and socioeconomic level are consistently associated with a higher risk of developing RA [6]. It's important to emphasize that one's diet significantly influences the makeup of their microbiota, which has been linked to the disease's onset and progression (Figure 2).

**Figure 2:** The involvement of diet in the development of rheumatoid arthritis (RA). Figure credit: Author (Kartikey Vats Shekhar) TMAO: Trimethylamine N-oxide

Smoking

Compared to women, men seem to face a higher level of risk than women of getting RA due to smoking. Remarkably, if you stop smoking, the correlation between your chances of developing RA seems to decrease. To be more precise, the correlation between smoking and the risk of anti-citrullinated peptide antibody-negative RA (ACPA-negative RA) vanished entirely twenty years after stopping. In contrast, the correlation with the risk of ACPA-positive RA remained linked to the quantity of cigarettes smoked. The connection between smoking and the widely recognized genetic susceptibility marker, known as the HLA-DRB1 SE, and how this association impacts the onset of RA in individuals with both antibody-positive and antibody-negative forms is a subject of interest [7]. Smokers with two copies of the SE had a 21-fold increased risk of getting RA compared to non-smokers without any SE copies. Furthermore, the quantity and severity of smoking raised the likelihood of ACPA-positive RA linked to SE and smoking. In the context of ACPA-positive RA, our findings highlight a strong gene-environment interaction and a dose-response connection between genetic and environmental risk variables [8].

RETRACTED

Silica

Exposure to silica is the second most commonly stated environmental risk linked to the onset of RA. Despite accounting for the influence of smoking, various longitudinal and case-control investigations have uncovered associations between RA in males and specific occupations, including those involving granite workers, rock drillers, and stone crushers. Notably, case-control studies have revealed an inverse relationship between silica exposure and the risk of RA in individuals working with sandstone, ceramics, and refractory materials. Like smoking, silica exposure is largely linked to seropositive RA [9]. Interestingly, smokers exposed to silica had a significant incidence of ACPA-positive RA, suggesting that these exposures may interact. But, as these results don't account for variables like duration or intensity, care should be exercised when interpreting them [10].

Reproductive factors in women

Studies investigating the complex and multifaceted pathophysiology of RA have emphasized the role of female hormones, including progestogens and estrogen.

Gender Discrepancy

Before age 50, the ratio of women to men diagnosed with RA was 2:4, indicating a higher prevalence in women. This suggests that female hormones may play a role in susceptibility.

Age-Related Shifts

Beyond 60, the proportion of women to men decreases, suggesting that the impact of female hormones on RA risk may vary with age [11].

Postpartum and Menopause

Given the elevated prevalence of RA during these life stages, it's conceivable that hormonal changes associated with these transitions contribute to the onset of the condition.

Reproductive Years

Approximately 50% of RA cases initiate during a woman's reproductive years, implying a potential connection between the disease's development and female hormones.

RETRACTED

Hormonal Fluctuations

Changes in hormonal exposure in females, as seen in events like pregnancy, postpartum, breastfeeding, menopause, and the utilization of external hormones, can induce fluctuations in their hormonal profiles. It is crucial to note that the impact of female hormones on RA can exhibit both pro-inflammatory and anti-inflammatory characteristics. This duality is contingent upon factors like serum hormone concentrations and the particular stage of the reproductive cycle. Ongoing research is actively investigating the precise mechanisms by which these hormones impact the pathophysiology of RA. While these findings suggest a link between female hormones and RA, rheumatologists diligently study the exact role and underlying mechanisms [12].

Impacts of body composition on RA

An individual's body composition can majorly impact how likely they are to develop RA. Obesity, a higher body mass index (BMI), and an enlarged waist measurement are risk factors for RA. Because white adipose tissue may create pro-inflammatory mediators, including IL-6, interferon (IFN)-alfa, C-reactive protein (CRP), and adipokines, it is classified as an "endocrine organ." The heightened synthesis of pro-inflammatory substances promotes the onset of autoimmunity. Leptin is an inflammatory adipokine that inhibits regulatory T-cell function in addition to inducing the production of inflammatory cytokines by macrophages. Leptin hormone hinders B-cell apoptosis and increases autoreactive cell preservation and growth in the preclinical stage of RA. Another adipokine that has several uses and structural similarities to tumor necrosis factor-alpha (TNF-α) is called adiponectin [13]. In people with RA, adiponectin contributes to the inflammatory environment that fosters osteoclast formation in the synovial tissue. A disease known as "sarcopenic obesity," which affects up to two-thirds of people with established RA, especially women, is typified by a rise in fat mass and muscle atrophy without a discernible change in body weight. Pro-inflammatory cytokines found in skeletal muscles encourage the breakdown of muscle proteins and cause a decrease in muscle mass. Nonetheless, several lifestyle choices, such as glucocorticoid usage, food habits, and inactivity greatly increase the likelihood of RA patients acquiring sarcopenic obesity [14]. 

Elimination diet

Rheumatoid arthritis symptoms might be made worse by several meals and dietary ingredients. An "elimination diet" strategy, which involves removing food-related antigens that may exacerbate illness symptoms, may thus be taken into consideration [15]. The mucosal immune system and the external environment are shielded from one another by the intestinal epithelium. The immunological response that develops in response to certain food antigens is largely determined by this barrier [16]. Several investigations have suggested that some foods may function as antigens in the human body. They pass through the epithelium of the gastrointestinal tract, engage the mucosal immune system, and then reach the circulation. Additionally, it has been noted that the gut mucosa of RA patients on non-steroidal anti-inflammatory drugs (NSAIDs) becomes more permeable to allergens [17]. Two groups of RA patients who tested positive for the antibody were included in the research. While the other group had a diet confined to allergies, including lactoproteins and yellow colors, the first group abstained from additives, allergens, and preservatives. Patients with RA who adhered to these dietary plans achieved similar clinical outcomes [18].

RETRACTED

Two groups of RA patients were included in another study by Karatay et al.: those with a positive skin prick test (SPT) reaction to a minimum of one food item and those having wholly negative SPT findings. Every patient adhered to an exclusion diet for a certain amount of time. Foods that produced positive skin prick reactions were given to the Patient Participation Group (PPG), whereas larger amounts of highly allergic maize and non-allergenic rice- known to cause allergies in RA patients were ingested by the placebo non-allergenic grain (PNG) group. This was followed by a re-elimination phase [19]. Many indicators showed increases during and after the re-elimination phase among the PPG, including Erythrocyte Sedimentation Rate (ESR), CRP, pain, joint swelling, joint sensitivity, Risk Analysis Index (RAI) score, TNF, and IL-1. According to these studies, food allergies could work as immune system triggers, causing macrophages and other effector cells to become active and causing inflammation. In RA therapy, inflammatory mediators such as TNF-α and IL-1 are addressed. Interestingly, eating foods that trigger allergies seems to increase these inflammatory mediators. Thus, cutting out certain items that cause allergies from RA patients' diets could be advantageous, perhaps lessening the requirement for anti-TNF-α and recombinant human IL-1 receptor antagonists throughout their therapy [20].

Dietary fibres and whole grains

Previous studies have established a clear inverse correlation between the consumption of dietary fiber and markers of inflammation, such as plasma fibrinogen, TNF-α, high-sensitivity CRP (hs-CRP), and IL-6 levels, which are indicative of rheumatoid arthritis [21]. Food items are considered "whole" when they contain equal amounts of germ, endosperm, and bran, akin to whole grains. Whole cereals like wheat, corn, rye, whole rice, oats, barley, millets, sorghum, canary seed, fonio, and wild rice are renowned for their high levels of antioxidants, phytic acid, vitamin E, and selenium. These constituents are believed to contribute to reducing inflammation [22]. The Food and Drug Administration (FDA) has authorized claims for health promotion regarding dietary fibers and whole grains in relation to RA, even in the absence of conclusive evidence. As per the Dietary Reference Intakes recommendations, a dietary fiber intake within the range of 14 grams per 1,000 kilocalories, or 25 grams for adult women and 38 grams for adult men, is deemed beneficial for one's health [23].

RETRACTED

Spices

Due to strong phenolic compounds, including shogaols and gingerols, ginger has long been known for its medicinal benefits. Turmeric, abundant in phenolic curcuminoids, has also demonstrated anti-tumor properties [24]. In research, the adjuvant-induced arthritic rats received a precise combination of ginger and turmeric. This combination showed protective benefits against RA extra-articular complications. In a separate research, the same team discovered that ginger and turmeric, when combined at a dose of 200 mg/kg body weight, might independently reduce RA signs and symptoms in male Wistar albino rats that had been subjected to an adjuvant-induced arthritic condition. The results demonstrated statistical significance, as evidenced by a p-value of 0.05 when compared to the control group that solely received indomethacin [25].

In an in vitro investigation using synoviocytes generated from RA patients and expressing IL-1 and IL-6, curcumin has also been demonstrated to be a strong anti-inflammatory spice [26]. For the treatment of RA, methotrexate is a commonly used antirheumatic medication; however, it also causes vascular endothelial dysfunction and elevates oxidative stress. Methotrexate-induced vascular endothelial dysfunctions in male Wistar rats were reported to be reduced by co-administration of curcumin and folic acid [27]. In many Southeast Asian cuisines, cinnamon bark, or *Cinnamomum zeylanicum*, is employed. The polyphenolic fraction of cinnamon bark was used by Rathi et al. to treat male Swiss albino mice and Wistar rats used as RA animal models. In their research, it was found that there were inhibitory effects observed in the release of cytokines such as IL-2, IL-4, and IFN, along with a reduction in TNF-α levels [28].

Essential fatty acids

The ability of omega-3 or omega-6 fatty acids to reduce inflammation and inhibit the immune system has been demonstrated. Gamma-linolenic acid (GLA), an omega-6 fatty acid, is abundant in borage seed oil. Thirty-seven patients with active RA participated in a double-blind experiment where they were given borage seed oil containing 1.4 g of GLA daily, whereas the placebo group received cottonseed oil. The group that got GLA had considerably lower ratings for sore and swollen joints after 24 weeks of intake, whereas the placebo group showed no change [25]. The medicinal potential of gamma-linolenic acid, omega-3 fatty acids alpha-linolenic and stearidonic acid, and black currant seed oil (BCSO) has also been studied. In a double-blind study, RA patients received 10.5 g of BCSO and soybean oil as a placebo for 24 weeks. Compared to the placebo group, the BCSO-treated group showed significantly better results regarding joint tenderness and pain relief [29].

RETRACTED

High levels of omega-3 fatty acids are found in fish oils, and several controlled studies have examined how well they work to treat RA. In a double-blind study, RA patients were given fish oil containing 3.6 g of omega-3 fatty acids daily. At the same time, the placebo group received a combination of fatty acids for 12 weeks, comparable to the amount found in a typical diet. Compared to the placebo group, the fish oil group had less morning stiffness and a notable gain in grip strength. The capacity of the omega-3 fatty acids eicosapentaenoic and docosahexaenoic acids to lessen the severity of RA has been studied. Compared to the placebo group, which got just maize oil, RA patients who took these derivatives in a dose of 130 mg/kg body weight/day for 26-30 weeks experienced significantly less discomfort, morning stiffness, and painful joints [30].

Alcohol

There is ongoing discussion over the connection between alcohol use and the onset of RA. While some studies suggest that drinking alcohol might accelerate the course of RA, other studies find no evidence of this relationship. Alcohol usage was shown to be dose-dependently related to a lower incidence of RA as compared to non-drinkers in a recent case-control research conducted in a Scandinavian population. These results were consistent with gender, age, and variations in cyclic citrullinated peptide (CCP) status [31]. In another study, which concentrated on the frequency of alcohol intake among Caucasian RA patients rather than the quantity, a similar tendency was seen. Researchers found a notable inverse correlation between increased alcohol consumption and the severity indicators of RA, encompassing factors such as CRP levels, the Disease Activity Score in 28 joints (DAS28), the modified Health Assessment Questionnaire, and the Pain Visual Analog Scale (VAS).

RETRACTED

Tea

The natural substance epigallocatechin-3-gallate (EGCG), which is gaining much interest as a nutraceutical, has demonstrated encouraging therapeutic qualities. Extracted from the dried leaves of *Camellia sinensis* and *Camellia assamica*, two members of the Theaceae family of plants, it is the primary phytochemical in green tea. The prophylactic properties of green tea against a range of maladies, such as neurological diseases, inflammatory disorders, cardiovascular ailments, and various malignancies, have been extensively demonstrated [32]. The resistance of synovial fibroblasts to apoptosis is one of the unique characteristics of RA. This resistance is frequently associated with the overexpression of anti-apoptotic proteins such as Mcl-1 and B-cell lymphoma-2 (Bcl-2) and the ongoing synthesis of proteins like nuclear factor (NF) and protein kinase B (PKB). Research has effectively demonstrated that synovial fibroblasts' Mcl-1 levels may be lowered by EGCG injection, increasing the cells' susceptibility to apoptosis. Furthermore, EGCG effectively inhibits the synthesis of matrix metalloproteinases (MMP-1, MMP-2, and MMP-3) in synovial fibroblasts, thereby halting the degradation of bone and cartilage. EGCG therapy reduces the production of IL-1 and IL-6 by synovial fibroblasts in RA patients while enhancing the activity of the soluble glycoprotein gp130 receptor inhibitor, which in turn inhibits IL-6 trans-signaling [33].

Red meat

The first research to look at the relationship between eating red meat and the likelihood of developing inflammatory polyarthritis was conducted by Pattison et al. [34]. According to their research, consuming more red meat and protein may raise your chance of developing inflammatory polyarthritis. They did admit, though, that it was unclear whether these correlations resulted from other lifestyle variables or causal. Later, several prospective cohort studies investigated the association between meat consumption-including red meat, processed meat, and poultry, and the chance of developing RA. Still, none of them found a statistically significant correlation [35].

Gluten

Gliadin and glutenin, the main proteins in wheat grains, form a complex combination called gluten, which can cause an immunological reaction, particularly in celiac disease patients. According to recent studies, gluten may also function as an antigen in RA, changing the immune system's response [36]. A year of strict adherence to a vegan, gluten-free diet was associated with a substantial drop in antibodies against gliadin and beta-lactoglobulin and a decline in the incidence of disease in individuals with RA. Lower levels of low-density lipoprotein (LDL) and oxidized LDL were seen in another randomized research with 66 RA patients who followed the same dietary pattern, which similarly showed protective benefits against atherosclerosis and inflammation [37].

RETRACTED

Fasting

Subtotal fasting involves a restricted intake of carbohydrates and energy, primarily through vegetable juice and vitamin and mineral supplements. Fasting can reverse the usual immunological condition associated with RA by lowering the quantity and activity of CD4+ cells. Increased Th1 and Th17 lineage differentiation and activation of CD4+ T cells are common in RA [38]. T cell activation can be reduced by a brief (7-10 days) fasting period, which can also have a transient immunosuppressive impact. While evidence of decreased pain and inflammation (as assessed by ESR and CRP) has been shown while fasting, these benefits are transient and do not result in long-term adjustments to disease activity [39].

Vegan diet

It has been demonstrated that a vegan diet, rich in dietary fibers, lactobacilli, and antioxidants, can improve the composition of the gut flora and RA disease activity. Twenty-four people with moderate to severe RA participated in a single-blind dietary intervention experiment and followed a low-fat diet (less than 10% fat) for four weeks. Except for the length of the morning stiffness, there were notable decreases in body weight and RA symptoms after this time [40]. A comparative analysis of all the studies included in the review is described in Table 1.

**Table 1:** Comparative analysis of all the studies included in the review.

Author	Journal and year of publication	Inference
Aletaha D, et al. [1]	Arthritis Rheum, 2010	A novel classification system shifts the focus in rheumatoid arthritis (RA) from late-stage features to early-stage indicators of persistent and erosive disease, emphasizing the urgency of early diagnosis and effective treatment to mitigate undesirable consequences.
Cobb S, et al. [2]	N Engl J Med, 1953	Rheumatoid arthritis patients in this study had higher mortality rates, especially among younger males, primarily due to causes like valvular heart disease, infections, renal disease, and pulmonary embolism, while certain causes were less frequent. Further research is needed for detailed analysis.
Klockars M, et al. [3]	Br Med J Clin Res Ed, 1987	A Finnish study on granite workers observed higher rates of disability pensions and free medicine use for rheumatoid arthritis compared to the general male population. The RA cases among workers were often severe, seropositive, and erosive, possibly linked to quartz exposure's immune system effects.
Del Rincón ID, et al. [4]	Arthritis Rheum, 2001	Rheumatoid arthritis (RA) patients face a higher risk of cardiovascular events beyond traditional risk factors, highlighting the need for RA-aware healthcare providers to adopt suitable diagnostic and therapeutic strategies.
Khan N, et al. [5]	Cancer Res, 2006	Cell signalling pathways are crucial in balancing cell growth and death, making them attractive targets in cancer management. Green tea, particularly epigallocatechin-3-gallate (EGCG), shows promise in cancer prevention and therapy by influencing these pathways. This review explores EGCG's impact on cancer management through signaling pathway modulation.
Scher JU, et al. [6]	Elife, 2013	Rheumatoid arthritis (RA) results from genetic and environmental factors. Study links *Prevotella copri* in the gut to new-onset untreated RA patients, potentially influencing disease development and gut microbiota balance.
Krause D, et al. [7]	Arthritis Rheum, 2000	Severe rheumatoid arthritis (RA) patients unresponsive to methotrexate (MTX) treatment face a significantly elevated mortality risk, over 4 times higher than the general population, in contrast to MTX-responsive RA patients with a more modest increase in mortality.
Chen J, et al. [8]	Genome Med, 2016	Imbalances in the gut microbiota in rheumatoid arthritis (RA) patients may stem from overrepresenting specific, uncommon bacterial lineages. Understanding the link between gut microbiota and metabolic markers could help predict RA development and progression.
Raghav SK, et al. [9]	Mediators Inflamm, 2006	In rheumatoid arthritis (RA) patients, peripheral blood mononuclear cells (PBMCs) displayed increased expression of tumor necrosis factor-alpha (TNF-α) and tumor necrosis factor receptor 1 (TNFR-I), alongside elevated levels of signaling intermediates TRADD, RIP, and TRAF-2, indicating augmented TNF-α signaling pathways in RA. However, additional regulatory mechanisms are likely at play.
Ajeganova S, et al. [10]	Arthritis Care Res, 2013	Obesity in rheumatoid arthritis (RA) is linked to poorer disease outcomes and increased comorbidities. The use of body measurements is advised to enhance the prediction of RA's progression.
Gorvitovskaia A, et al. [11]	Microbiome, 2016	The term "enterotypes" is deemed misleading, as it suggests consistent community taxa and distinct human gut sample groupings, which do not align with the broader data. "Biomarker" is suggested as a more accurate descriptor for taxa correlating with diet, lifestyle, and disease.
Bernard NJ [12]	Nat Rev Rheumatol, 2014	Researchers identified a high prevalence of *Prevotella copri *in rheumatoid arthritis (RA) patients, particularly those with new-onset untreated RA (NORA). They detected a potential link between *P. copri* and RA, but more research is needed to establish causation and mechanisms.
Maeda Y, et al. [13]	Arthritis Rheumatol, 2016	Dysbiosis was shown to enhance arthritis susceptibility by activating self-targeting T cells in the gut. In mice, dysbiotic gut microbiota triggered joint inflammation, highlighting its role as an environmental factor in arthritis development.
Chiang HI, et al. [14]	J Clin Med, 2019	In rheumatoid arthritis (RA), gut microbiota composition differed from healthy controls. RA patients had reduced diversity, increased Verrucomicrobiae, and specific bacterial associations with inflammatory markers and auto-antibodies, supporting gut microbiota's role in RA development.
Rubbert-Roth A, et al. [15]	Arthritis Res Ther, 2009	Rheumatoid arthritis is primarily treated with conventional drugs like methotrexate. TNF inhibitors are effective but not for all. Patients with inadequate responses have options, including switching to different biologics like rituximab and abatacept.
Jacobsson LT, et al. [16]	BMJ, 2003	The presence of older siblings was linked to a higher risk of ankylosing spondylitis (AS). Further studies in different populations are necessary to validate these findings.
Edwards CJ [17]	J Rheumatol, 2008	Rheumatoid arthritis results from genetic and environmental factors, with recent research indicating gut microbiota differences in RA patients. Mechanisms linking gut bacteria to RA and treatment effects require further study. Understanding gut bacteria's impact on immune function and inflammatory joint diseases is crucial.
Eggert M, et al. [18]	Curr Pharm Des, 2010	Autoantibodies are prevalent in autoimmune diseases like rheumatoid arthritis (RA), systemic lupus erythematosus (SLE), and multiple sclerosis (MS). While they aid in diagnosis and prognosis for RA and SLE, no specific antibody is exclusive to MS. Monitoring autoantibody levels in RA and SLE can help assess therapy response, mainly when using costly biological treatments.
Yahya A, et al. [19]	Mod Rheumatol, 2014	In the Malaysian genetic context, exposure to silica and cigarette smoke increases the risk of developing rheumatoid arthritis (RA). This research connects environmental lung exposures and anti-citrullinated peptide antibody (ACPA)-positive RA in Asian populations.
Stolt P, et al. [20]	Ann Rheum Dis, 2010	Among men, the combination of silica exposure and smoking elevates the risk of developing ACPA-positive RA. This implies that various inhalation exposures might interact in the development of ACPA-positive RA.
Sankrityayan H, et al. [21]	Can J Physiol Pharmacol, 2016	Chemotherapy is an essential cancer treatment, but it often leads to severe side effects. Curcumin, a compound from the plant *Curcuma longa L.*, shows promise in preventing and reducing chemotherapy-induced side effects, protecting normal cells and enhancing cancer cell sensitivity to treatment.
Zeng L, et al. [22]	Transplant Proc, 2008	This study investigates the role of Roundabout 4 (Robo4) in protecting microvascular endothelial cells from irradiation-induced damage. Robo4 helps maintain endothelial integrity, preserves junctional molecules, and reduces permeability.
Kloesch B, et al. [23]	Int Immunopharmacol, 2013	Curcumin, a natural compound, displays potent anti-inflammatory effects and promotes apoptosis in fibroblast-like synoviocytes (FLS). This research highlights its potential as a natural remedy for chronic inflammatory diseases, including rheumatoid arthritis (RA).
Gioia C, et al. [24]	Nutrients, 2020	RA's development involves genetic and environmental factors. Diet plays a role in RA risk, impacting gut microbiota and body composition. Nutrients like those in the Mediterranean diet, vitamin D, and probiotics could complement standard RA treatments, emphasizing the significance of a healthy lifestyle and nutrition for RA patients.
Alamanos Y, et al. [25]	Autoimmun Rev, 2005	Rheumatoid arthritis (RA) varies globally, with higher prevalence in Northern European and North American regions. Genetic, environmental, and lifestyle factors, including genetics, age, gender, smoking, and more, contribute to RA's risk and severity.
Wang H, et al. [26]	Biomed Chromatogr, 2014	Huo Luo Xiao Ling Dan (HLXLD), a traditional Chinese herbal formula for arthritis, was studied for its pharmacokinetics compared to *Boswellia serrata* extract in normal and arthritic rats. Results showed improved absorption in HLXLD, suggesting a synergistic effect of its herbal ingredients for enhanced efficacy.
Ammon H [27]	Wien Med Wochenschr, 2002	*Boswellia serrata* gum resin, a traditional remedy in Ayurvedic medicine, contains boswellic acids pentacyclic triterpenes with genuine anti-inflammatory effects. They inhibit leukotriene biosynthesis, induce apoptosis, and impact various inflammatory diseases like rheumatoid arthritis, colitis, and bronchial asthma. Clinical trials have shown promise in these conditions.
Rathi B, et al. [28]	Sci Pharm, 2013	The study evaluated the effectiveness of a polyphenol fraction from Cinnamomum zeylanicum bark (CPP) in various animal models of inflammation and arthritis, showcasing a dose-dependent reduction in paw swelling, reversal of weight loss in induced edema, and a significant decrease in TNF-α levels without causing gastric issues. These findings suggest that CPP exhibits strong potential as an anti-rheumatic agent with disease-modifying properties, demonstrating notable action in alleviating inflammation and arthritis in animal models.
Ahmed S, et al. [29]	Arthritis Rheum, 2006	EGCG, a compound found in green tea, demonstrated the ability to inhibit the production of inflammatory molecules and enzymes in rheumatoid arthritis synovial fibroblasts. This suggests its potential as a therapeutic agent for preventing joint damage in RA.
Clement Y [30]	Prev Med, 2009	While clinical evidence is not definitive, regular consumption of green tea shows potential for preventing prostate and breast cancer. It may also help reduce the risk factors associated with atherosclerosis and lower the incidence of cardiovascular events and strokes.
De Santis S, et al. [31]	Front Immunol, 2015	The intestinal tract acts as a critical interface between the external environment and the body. It regulates responses to dietary antigens to prevent damage. This review explores how dietary components and microbiota affect the intestinal barrier and permeability and their potential impact on health and treatments.
Mu Q, et al. [32]	Front Immunol, 2017	Intestinal epithelial barrier integrity is crucial in preventing a "leaky gut." Dysregulation can trigger autoimmune diseases. Probiotics and antibiotics show promise in modulating the gut microbiota to regulate permeability and potentially mitigate autoimmune diseases.
Van Spaendonk H, et al. [33]	World J Gastroenterol, 2017	The gastrointestinal barrier, vital for nutrient absorption and antigen exclusion, relies on intercellular junction proteins. Excessive protease activity contributes to increased permeability and is associated with various diseases, suggesting potential therapeutic targets.
Pattison DJ, et al. [34]	Arthritis Rheum, 2004	A high level of red meat consumption may represent a novel risk factor for inflammatory arthritis or may act as a marker for a group of persons with an increased risk from other lifestyle causes.
Noonan CW, et al. [35]	Environ Health Perspect, 2006	Initial results suggest a connection between asbestos exposure and systemic autoimmune diseases (SAID). Further investigation with precise exposure measurements will provide more insights into this potential association.
Lundberg I, et al. [36]	Scand J Rheumatol, 1994	This Swedish study of 500,000 individuals assessed RA incidence across various occupations and exposures, revealing slight risk variations. Some jobs, like cost accountants, showed higher RA risk, while farmers and concrete workers displayed increased risk despite potential selection bias. Substantial organic solvent handling, as indicated by a job-exposure matrix, was also associated with greater relative risk.
Reckner Olsson Å, et al. [37]	Scand J Work Environ Health, 2000	While many findings align with prior research, this study reveals novel associations between increased rheumatoid arthritis risk and asphalt workers and service station employees not previously reported in the literature.
Grant WB [38]	Br J Nutr, 2000	This review discusses the links between dietary components and rheumatoid arthritis (RA). It highlights the potential role of meat and offal consumption, particularly their fat content, in contributing to RA-related inflammation.
Costenbader KH, et al. [39]	Am J Epidemiol, 2010	This study investigated the relationship between antioxidant intake, including vitamins A, C, E, and various carotenoids, and the risk of developing rheumatoid arthritis and systemic lupus erythematosus. The results showed no significant associations between antioxidant intakeand the risk of these autoimmune diseases in women.
Manzel A, et al. [40]	Curr Allergy Asthma Rep, 2014	In developed societies, lifestyles, and dietary patterns, particularly the "Western diet" rich in fats, sugars, and processed foods, contribute to the rise of metabolic, cardiovascular, and autoimmune diseases. T cells play a crucial role in connecting dietary factors to autoimmunity.

RETRACTED

## Conclusions

In conclusion, eating a diet high in raw or mildly cooked vegetables, especially greens and legumes, as well as adding spices like ginger and turmeric, might be beneficial for treating rheumatoid arthritis (RA). The diet should also include seasonal fruits and probiotic yogurt, which are high in natural antioxidants and anti-inflammatory qualities. On the other hand, meals heavy in salt, oils, butter, sugar, and animal products should be avoided by patients, as well as processed foods. Furthermore, nutritional supplements such as multivitamins, vitamin D, and cod liver oil can help treat RA. This dietary-focused strategy and low-impact aerobic training can be utilized to improve RA self-management at a reasonable cost. Nevertheless, it's important to emphasize that great patient compliance is usually required for effective RA therapy and management. Studies have repeatedly shown that smoking greatly increases the chance of RA, especially in those genetically predisposed to the condition. Exposure to silica is a strong non-smoking inhalant risk factor for RA, and it may interact with smoking. These two variables are linked to a common notion of systemic and pulmonary mucosal inflammation. Among the other inhalants, silica is the most significant inhalant risk factor. Though several research have examined possible links between different reproductive variables and the risk of RA, the impact of female hormones on that risk is still unknown. Inconsistent findings might be ascribed to methodological flaws and biases, including failing to account for smoking. Higher hormonal levels are associated with factors like early menarche, late menopause, parity, postmenopausal hormone therapy (PMH), and oral contraceptive use; lower hormonal levels are associated with postpartum status, early menopause, late menopause, and the use of anti-estrogen medications. A fascinating method for researching hormone exposures in females may be to evaluate total hormonal exposures while considering a woman's lifetime reproductive experiences.
